RETRACTED

# Rehmannia Glutinosa Extract Activates Endothelial Progenitor Cells in a Rat Model of Myocardial Infarction through a SDF-1 α/CXCR4 Cascade

**DOI:** 10.1371/journal.pone.0054303

**Published:** 2013-01-18

**Authors:** Ying-Bin Wang, Yun-Fang Liu, Xiao-Ting Lu, Fang-Fang Yan, Bo Wang, Wen-Wu Bai, Yu-Xia Zhao

**Affiliations:** 1 Key Laboratory of Cardiovascular Remodeling and Function Research, Shandong University, Jinan, Shandong, China; 2 Department of Traditional Chinese Medicine, Qilu Hospital, Shandong University, Jinan, Shandong, China; 3 Department of Diagnosis, College of Medicine, Shandong University, Jinan, Shandong, China; National Cancer Institute, United States of America

## Abstract

**Objectives:**

Endothelial progenitor cells (EPCs) can be used to repair tissues after myocardial infarction (MI) but EPC activators have adverse reactions. Rehmannia glutinosa is a herb used in traditional Chinese medicine, which can promote bone-marrow proliferation and protect the ischemic myocardium. We investigated the effects of Rehmannia glutinosa extract (RGE) on EPCs in a rat model of MI.

**Methods:**

A total of 120 male Wistar rats were randomized to 2 groups (n = 60 each) for treatment: high-dose RGE (1.5 g·kg^−1^·day^−1^ orally) for 8 weeks, then left anterior descending coronary artery ligation, mock surgery or no treatment, then RGE orally for 4 weeks; or normal saline (NS) as the above protocol. The infarct region of the left ventricle was assessed by serial sectioning and morphology. EPCs were evaluated by number and function. Protein and mRNA levels of CD133, vascular endothelial growth factor receptor 2 (VEGFR2), chemokine C-X-C motif receptor 4 (CXCR4), stromal cell–derived factor-1α (SDF-1α) were measured by immunohistochemistry, Western blot and quantitative PCR analysis.

**Results:**

RGE significantly improved left ventricular function, decreased the ischemic area and the apoptotic index in the infarct myocardium, also decreased the concentration of serum cardiac troponin T and brain natriuretic peptide at the chronic stage after MI (from week 2 to week 4). RGE increased EPC number, proliferation, migration and tube-formation capacity. It was able to up-regulate the expression of angiogenesis-associated ligand/receptor, including CD133, VEGFR2 and SDF-1α/CXCR4. In vitro, the effect of RGE on SDF-1α/CXCR4 cascade was reversed by the CXCR4 specific antagonist AMD3100.

**Conclusion:**

RGE may enhance the mobilization, migration and therapeutic angiogenesis of EPCs after MI by activating the SDF-1α/CXCR4 cascade.

## Introduction

Myocardial infarction (MI) occurs with the deprivation of coronary blood and is usually caused by stenosis or occlusion of the coronary artery. The culminating event is necrosis of myocardial tissue and dysfunction of the left ventricle. Bone-marrow-derived stem cells, including endothelial progenitor cells (EPCs), are attractive targets for repair of the ischemic myocardium [1]–[3]. EPCs can home to ischemic tissues and contribute to therapeutic angiogenesis [4]–[5]. Many EPCs agonists such as granulocyte-colony stimulating factor, vascular endothelial growth factor (VEGF) and statins, can mobilize EPCs in bone marrow [6]–[7]. However adverse reactions, such as increased vascular permeability and high ratio of restenosis and liver damage, limit their use for MI [8]. A safe EPC activator is needed for MI therapy.

RETRACTED

Activated EPCs first migrate to the ischemic tissue for their roles. Stromal-derived factor-1 (SDF-1, or CXCL12) is the only known chemokine capable of migration of hematopoietic stem cells (HSCs), as the fluctuations in SDF-1 expression controlled the fluctuated steady-state of HSCs and their progenitors in peripheral blood [9]. Among these, the SDF-1α and its receptor 4 (CXCR4) play a key role in mobilization and migration of EPCs [10]. After MI, SDF-1α/CXCR4 interaction plays a crucial role in recruiting EPCs to the ischemic myocardium, the increased CXCR4 expression lead to increased EPCs homing to the ischemic zone and participated in therapeutic angiogenesis [11]–[13]. These suggest that the SDF-1α/CXCR4 cascade is critical for the regulation of EPCs, and it might be an important therapeutic target for cardiovascular diseases especially in MI [14].

Rehmannia glutinosa, belongs to the family of Scrophulariaceae, is a widely used traditional Chinese medicinal herb. It has been used to treat hypodynamia caused by many kinds of diseases for thousands of years in China, Japan, Korea and many other Asian countries. It has been effective and safe, but the involved mechanism has not been verified. Recently, Rehmannia glutinosa extract (RGE) has been used in modern medicine studies [15]. RGE can stimulate the proliferation and differentiation of hematopoietic stem cells in bone marrow [16] and increase the numbers of leucocytes, thrombocytes, reticulocytes and DNA content of bone marrow [17]. Furthermore, RGE can antagonize myocardial cell death induced by caspase-3 activation, thus protecting the ischemic myocardium [18].

Our preliminary experiments in rat showed an increase in number of EPCs in blood and bone marrow after oral administration of RGE (Table S1). These suggested that RGE had effect on EPCs.

In this study, we used the rat MI model to imitate the pathological changes after MI and observed the effects of RGE on preserving the left ventricle, up-regulating the number and function of EPCs and increasing therapeutic angiogenesis. Thus, we could examine whether the RGE is a EPCs activator or not. We further analyzed the alteration of the SDF-1α/CXCR4 cascade with RGE in vivo and in vitro, to investigate the possible mechanism of RGE on EPCs after MI.

RETRACTED

## Materials and Methods

### Preparations of Rehmannia Glutinosa Extract (RGE)

Rehmannia glutinosa (purity>96%) was from the National Institutes for Food and Drug Control (Beijing). RGE was prepared by alcohol extraction. Briefly, dried Rehmannia glutinosa was soaked with distilled water in a 1∶10 volume ratio for 24 h, then heated to 80°C for 12 h. The supernatant was collected and ethanol was added to a 3∶4 volume ratio. The extracts were stored at room temperature for 24 h and centrifuged at 3000 rpm for 10 min, and the supernatant was mixed with ethanol in a 1∶4 volume ratio. Then extracts were incubated at room temperature for an additional 24 h and centrifuged at 3000 rpm for 10 min. Ethanol was evaporated from the supernatant. The extract was diluted in H_2_O and stored at 20°C overnight. This process was repeated 3 times. The final extracts were concentrated under reduced pressure and filtered, lyophilized, and serially stored at 4°C. The yield of dried extract (RGE) from starting crude materials was 22.5% (w/w) [19]. The RGE was dissolved in saline or phosphate-buffered saline (PBS) for experiments.

### Animal Models and Treatment

All animal surgeries were performed under isoflurane, and all efforts were made to minimize suffering.

A total of 120 male Wistar rats (Laboratory Animal Services Centre, College of Medicine, Shandong University; 8 weeks old; body weight 180 - 200 g) were fed a regular rat chow and housed in normal night-day conditions under standard temperature and humidity. All animal studies were carried out at the Animal Care Center of Key Laboratory of Cardiovascular Remodeling and Function Research, Shandong University. The experiment complied with the Animal Management Rule of the Ministry of Public Health, People’s Republic of China (document No. 55, 2001), and the experimental protocol was approved by the Animal Care Committee of Shandong University. The rats were randomly divided into 2 groups (n = 60 each) for treatment: control group, normal saline (NS) orally; treated group, high-dose RGE-NS solution of 1.5 g·kg^−1^·day^−1^ orally (in preliminary experiments, high-dose RGE, 1.5 g·kg^−1^·day^−1^ as compared with 0.38 and 0.75 g·kg^−1^·day^−1^, which was converted from human oral administration doses, effectively increased bone marrow mobilization of EPCs and migration to peripheral blood; TableS1). At the end of week 8, 20 rats from both groups underwent ligation of the left anterior descending coronary artery under endotracheal intubation and mechanical ventilation by use of the Harvard Appratus Mini-Vent (Type B-90218, China) [20]. Another 20 rats from both groups underwent mock surgery with a silk suture across the coronary artery without ligation. The other 20 rats in both groups were blank controls. The rats continued to be oral-fed RGE or NS, then rats were sacrificed, 5 each on the 3rd day and the end of 1, 2, 4 weeks, recording as day 3, week 1, week 2 and week 4 respectively.

RETRACTED

### Electrocardiography and Ultrasonic Cardiography

Before and after surgery, rats underwent electrocardiography (ECG) by use of a Micromaxx P04224 system (SonoSite, China) and ultrasonic cardiography (UCG) by a high-frequency duplex ultrasonic cardiogram system (Visual Sonics Vevo 770, Germany) and a transducer (RMV™ Scan Head 710B-048, Germany). Rats underwent ultrasonic cardiography at day 3, weeks 1, 2 and 4 before sacrificed. The transducer for ultrasonic cardiography was placed at the left thoraces between the 3rd and 4th ribs to obtain B-mode tracings of the heart from just below the level of the papillary muscles of the mitral valve. We obtained left-ventricular end-diastolic diameters (LVD-d) and end-systolic diameters (LVD-s) with M-mode tracings between the anterior and posterior walls. The time of end-diastole and end-systole was defined as time of maximum and minimum diameter of the left ventricle, respectively, in one heart cycle. Following the American Society of Echocardiology leading-edge method, we obtained 3 images, on average, in each view, which were averaged over three consecutive cycles [21].The system calculated the left-ventricular end-diastolic volume (LV-d), left-ventricular end-systolic volume (LV-s), mass of the left ventricle (LV-mass), left-ventricular fractional shortening (LVFS) and left-ventricular ejection fraction (LVEF).

### EPC Identification and Assessment of Function

#### Isolation and cultivation of EPCs

10 ml peripheral blood was obtained from rats by aspiration of the heart. Bone-marrow cells were obtained by flushing the cavity of femurs, tibias, and humerus with growth medium EBM-2 (Lonza Walkersville, USA, basal medium with 8 factors and 5% fetal bovine serum [FBS]). Peripheral blood and bone marrow mononuclear cells were isolated by Ficoll (Ficoll-Paque PLUS, GE Healthcare Bio-Sciences AB, USA) density-gradient centrifugation [22]. 10 million isolated cells were resuspended in growth medium EBM-2 and plated in 25-cm^2^ culture flasks. After 48 h, non-adherent cells were discarded and growth medium was changed every 2 days.

RETRACTED

#### Identification of EPCs

Direct fluorescent staining was used to detect dual binding of fluorescein isothiocyanate -labeled ulex europaeus agglutinin(FITC-UEA-1; Sigma, USA) and dioctadecyl-3,3,3′,3′-tetramethylindocarbocyanine-labeled acetylated low-density lipoprotein (Dil-acLDL; Invitrogen Molecular Probes, USA). Briefly, cells were incubated with Dil-acLDL (2 µg/ml) at 37°C for 2 h then fixed with 2% paraformaldehyde for 10 min. After a washing with PBS, cells were treated with FITC-UEA-1 (10 µg/ml) for 1 h. The nuclei were stained with 4′, 6-diamidino-2-phenylindole (DAPI) for viewing by laser scanning confocal microscope (LSMT10, ZEISS, Germany). Cells double stained for Dil-Ac-LDL and FITC-UEA-1 were considered EPCs [23]. Immunocytochemistry followed standard protocols.

#### Determination of EPC number

Fluorescence-activated cell sorting (FACS) was used to determine the EPC population in blood and bone marrow of rats. Briefly, fresh anticoagulation blood or bone-marrow PBS suspension (200 µl) was incubated with the monoclonal antibodies: anti-VEGFR2 (Abcam, USA, 1 mg/ml, 1∶100), anti-CD133 (Abcam, USA, 0.5 mg/ml, 1∶100) and anti-CD34-PerCP-Cy5.5 (Santa Cruz Biotechnology, Santa Cruz, CA; 0.2 mg/ml, 1∶10) for 20 min at room temperature, then with 2 ml Lysing solution (BD, USA) for 10 min and washed with PBS twice by centrifugation. The cells were resuspended with 200 µl PBS, then incubated with the secondary antibodies: goat polyclonal rabbit IgG-FITC (Abcam, USA, 2 mg/ml, 1∶80) and goat polyclonal mouse IgG-F(ab)2 fragment PE (Abcam, USA, 0.5 mg/ml, 1∶40) for 30 min at room temperature. Cells were washed with PBS and resuspended in 400 µl PBS. Flow cytometry involved use of a FACS calibur flow cytometer and Cell-Quest software (BD Biosciences, USA). Each analysis included at least 10,000 cells.

#### EPC proliferation, migration and tube formation

3-(4,5-dimethylthiazol-2-yl)-2,5- diphenyltetrazolium bromide (MTT) assay was used to evaluate EPC proliferation. Cells were cultivated for 4 days, then plated at 1×10^4^ per well in a 96-well plate with EBM-2 (200 µl) for 24 h. A filter-sterilized MTT solution was added for final concentration of MTT of 0.5 µg/ml for 4 h. The supernatant was discarded, and wells were washed twice with PBS. The EPC preparation was shaken at 90-100 rpm with 200 µl dimethyl sulfoxide for 10 min at room temperature. Optical density (OD) was measured at 490 nm. Each test was repeated 4 times [24].

EPC migration was evaluated by use of a transwell chamber (6.5 mm diameter inserts, 8.0 mm pore size; Corning, USA). Transwell inserts were placed in a 24-well plate containing EBM-2. EPCs (5×10^4^) were added to the upper chamber of the well, without FBS. Cells were allowed to migrate from the upper to the lower chamber for 12 h at 37°C. Non-migratory cells were removed from the upper chamber by wiping the upper surface with use of an absorbent tip. The number of migrating cells was counted in 5 different high-power fields per insert [25].

RETRACTED

Capillary-like tube formation was analyzed by use of Matrigel Matrix (BD Biosciences, USA). EPCs (8×10^4^ cells in 100 µl EBM-2) were placed in 96-well plates pre-coated with solidified Matrigel Matrix (100 µl) and cultured at 37°C for 24 h. Capillary-like tubular structures were photographed, and the number of incorporated EPCs in tubules was determined in 5 random fields. A tube was defined as a straight cellular segment connecting 2 cell masses (nodes) [26].

### ELISA

ELISA was used to measure cardiac troponin T (Tn-T) and brain natriuretic peptide (BNP) concentration in serum for left ventricular function evaluation, by use of a BNP kit (Rat-45, Abcam, USA) and Tn-T kit (TSZ ELISA, USA). Briefly, standards and diluted serum of rats were added into the pre-coated 96-well plates and incubated for 30 min in 37°C. After a washing with PBS, the horseradish peroxidase-conjugated anti-body was added for 30 min incubation at 37°C. After a washing by PBS, the tetramethylbenzibine substrate was added. After reaching the desired color density, the reaction was terminated by stop solution. OD_450_ was determined by use of an ELISA plate reader (Varioskan Flash, Thermo Fisher, Germany). Each samples repeated in 3 wells.

### Histology and Immunechemistry

Myocardial tissues (approximately 2 mm thick) in the left ventricle of rats were removed and fixed in 4% pre-cooled paraformaldehyde for 72 h, then embedded in paraffin, and sectioned into slices 5 µm thick. Poley’s stain was used to assess the ischemic myocardial area. Images were visualized under an optical microscope at ×200 magnification.

Myocardial tissue sections underwent the terminal deoxynucleotidyl transferase-mediated dUTP nick end-labeling (TUNEL) using an in situ detection kit (Roche, Germany) following the manufacturer’s instructions. The TUNEL apoptotic index was determined by calculating the ratio of TUNEL-positive cells to total myocardial cells.

Immunohistochemical staining involved standard techniques as described [27]. Briefly, endogenous peroxidase activity was inhibited by incubation with 3% H_2_O_2_. Sections were blocked with 5% calf serum in PBS and incubated overnight at 4°C with the monoclonal antibodies: anti-VEGFR2 (Abcam, USA, 1 mg/ml, 1∶100), anti-CD133 (Abcam, USA, 0.5 mg/ml, 1∶50) and anti-CXCR4 (Abcam, USA, 1 mg/ml, 1∶100). After a washing with PBS, sections were incubated with secondary antibody at 37°C for 30 min. Immunohistochemical staining was visualized by use of a diaminobenzidine kit (Zhongshan Goldenbridge Biotechnology, Beijing). Samples were counter stained with hematoxylin for nuclei.

RETRACTED

### RT-PCR

Tissue samples were frozen with the use of liquid nitrogen. Total RNA was extracted by use of TRIZOL reagent (Invitrogen, USA), quantified by spectrophotometry and reverse transcribed by use of the M-MLV Reverse Transcriptase System (Osaka, Japan) with oligo-dT primers. The mRNA expression of VEGFR2, CD133, and CXCR4 in myocardium was examined by real-time RT-PCR with SYBR Green Real-time PCR Master Mix (TOYOBO, Life Science Department, Japan) and an MYIQ™ Single Color Real-Time PCR Detection System (Bio-Rad, Germany). The mRNA sequences were obtained from Gene-bank (NCBI, Bethesda, MD; Table 1). Actin level was an internal control. Experiments were performed in triplicate, and data were analyzed by the 2^−△△CT^ method [28].

**Table 1:** Primers for RT-PCR.

Molecules	MW	Locus	Primer sequence	T_m_ °C
VEGFR2	123	NM_013062	F 5′-ATCGGTGAGAAAGCCTTGATCTC-3′	53
			R 5′-TTCTAGCTGCCAGTACCATTGGA-3′	
CD133	97	NM_001110137	F 5′-CTGCAAACCCATGATTACAGCAA-3′	57
			R 5′-CCCTATGCCGAACCAGAACAG-3′	
SDF-1α	240	NM_022177	F 5′-TCTTTGGCCTCCTGTAGAATGG-3′	56
			R 5′-TCACGGCAAGATTCTGGCTTA-3′	
CXCR4	177	NM_001033882	F 5′-CGTGAATGAGTGTCTAGGCAGG-3′	55
			R 5′-GGCTTTGGTTTTAAGTGCCATC-3′	
ACTIN	94	NM_0010822	F 5′-AGACCTTCAACACCCCAG-3′	55
			R 5′-CACGATTTCCCTCTCAGC-3′	

VEGFR2, vascular endothelial growth factor receptor 2; SDF-1α, stromal cell–derived factor-1α; CXCR4, chemokine (C-X-C motif) receptor 4; MW, molecular weight; T_m_, melting temperature.

### Western Blot Analysis

Total protein was isolated in lysis buffer (Beyotime, China) and was resolved by 10% SDS-PAGE, transferred to a nitrocellulose membrane, which was blocked in 5% skimmed milk in PBS containing 0.1% Tween-20 for 1 h at room temperature and incubated with monoclonal antibodies: anti-CXCR4 (Abcam, USA, 1 mg/ml, 1∶1000) and anti-SDF-1α(Abcam, USA, 0.5 mg/ml, 1∶500) overnight at 4°C. The bands were visualized with use of an enhanced chemiluminescence kit (Millipore, Billerica, MA, USA), photographed by use of Epson Perfection (V700 Photo, Japan) and analyzed by use of Quantity One software. Experiments were performed in triplicate, and data were normalized to level of β-actin.

### In vitro Cellular Experiments

To explore the molecular mechanism probably involved in the RGE effect on EPCs, EPCs from peripheral blood and bone marrow of normal rats were incubated in EBM-2 without FBS for 24 h. RGE was dissolved in PBS and filtered by millex (Millipore, USA, 0.22 µm), then added to EPCs at 10, 25, 50, 100, 500 and 1000 µg/ml. The inhibiter was CXCR4-specific antagonist AMD3100 (Abcam, USA; 5 µg/ml, purity >99%) for 1 h before RGE [29]. The blank control was cultivated with EBM-2.

RETRACTED

MTT was used to test proliferation of EPCs after stimulation for determining the proper concentration of RGE for EPCs. Western blot and real-time PCR analysis were used to examine the expression of SDF-1α/CXCR4 cascade in EPCs stimulated by RGE at different concentrations and for different time. Capillary-like tube formation was performed to test the function of RGE-stimulated EPCs.

### Statistical Analysis

Data are expressed as mean ± SD and were assessed by one-sample Kolmogorov–Smirnov test to check for normal distribution. Differences between 2 groups were assessed by unpaired *t*-test and among multiple groups by ANOVA followed by post-hoc two-tailed Newman-Keuls test. Data analysis involved use of SPSS 11.5 (SPSS Inc., Chicago, IL). Statistical significance was set at P<0.05.

## Results

During the experiment, 7 rats died: 2 each in the NS mock, NS MI and RGE MI groups and 1 in the RGE mock group.

### Model Evaluation and RGE’s Effect on the Improvement of Ischemic Myocardium

After surgery induction, the ECG revealed elevated ST segment and pathologic waveforms (Fig. 1-A), the UCG revealed changes in left ventricular wall mobility, blood flow at the mitral valve (Fig. 1-B) and the increased LV-d, LV-s, LV-mass, the decreased LVEF, LVFS, the reversed E/A ratio (P<0.01 to 0.05, Table 2 to 5). These revealed the successful establishment of the MI model. After MI, the function of left ventricular was reflected by LVEF of UCG. In acute stage (day 3 to week 1), the MI groups with both treatment showed almost no difference in LVEF, while as to the chronic stage (week 2 and week 4), the recovery of LVEF was greater with RGE than NS (P<0.05; Fig. 1-C). These revealed that RGE systemic delivery protected the function of left ventricular in chronic stage after MI.

**Figure 1:** Heart function and serum myocardium markers level of rats. (A) Electrocardiography (ECG) before and after myocardial infarction (MI). Leads I, II, III, aVR, aVL and aVF of normal (N) and MI rats. (B) Ultrasonic cardiography before and after MI. Images are M-mold (m) ultrasound and hemorheologic (h) ultrasound in normal and MI rats. (C) Left ventricular ejection fraction (LVEF) after MI. NS-b, normal saline (NS)-blank; NS-m, NS-mock; RGE-b, Rehmannia glutinosa extract (RGE)-blank; RGE-m, RGE-mock. (D) The levels of myocardium markers: cardiac troponin T (Tn-T) and brain natriuretic peptide (BNP). Data are mean ± SD. *P<0.05, **P<0.01 vs. NS group at the same time; ^#^P<0.05, ^##^P<0.01 vs. the same group at day 3.

RETRACTED

**Table 2:** UCE measurement before and 3 days after myocardium infarction (MI).

Group	LV,d (µl)	LV,s (µl)	LV,mass (mg)	LVEF (%)	LVFS (%)	E/A
NS-b prior	55.89±12.35	6.25±1.79	60.6±8.65	88.17±7.02	58.51±8.80	1.22±0.056
after	104.40±12.78	9.96±1.11	76.0±16.06	90.23±2.93	62.47±4.71	1.19±0.068
NS-m prior	105.00±42.34	8.44±2.11	80.10±13.62	90.82±5.61	63.41±9.38	1.21±0.096
after	185.60±33.83e	59.58±5.96	142.90±19.93e	67.76±3.22f	38.44±2.46f	1.10±0.058
NS-MI prior	98.98±5.59	10.38±0.82	72.00±9.38	89.52±1.68	61.05±2.28	1.22±0.059
after	440.30±51.03f	322.50±28.04f	315.20±60.45f	13.29±4.67f	26.97±8.93f	0.91±0.027f
RGE-b prior	108.50±28.67	13.25±1.05	74.14±7.59	87.52±1.58	57.49±2.46	1.14±0.045
after	119.30±10.59	22.56±3.22	65.45±8.55	81.12±5.82	50.38±5.72	1.18±0.056
RGE-m prior	94.63±17.94	11.62±2.61	67.66±7.48	87.99±5.19	58.67±7.46	1.16±0.071
after	109.80±5.50	29.36±2.54	115.10±31.00	73.32±2.95f	42.44±2.60e	1.16±0.048
RGE-MI prior	112.20±15.71	19.09±1.50	65.54±8.96	83.03±0.89	52.02±0.93	1.15±0.038
after	367.00±84.96f	234.30±38.74f	307.80±54.53f	19.01±6.86f	37.09±11.63e	0.81±0.147f

**Table 3:** UCE measurement before and 1 week after MI.

Group	LV,d (µl)	LV,s (µl)	LV,mass (mg)	LVEF (%)	LVFS (%)	E/A
NS-b prior	101.90±8.24	14.08±1.54	78.37±5.59	86.13±3.64	55.83±4.55	1.18±0.052
after	124.10±20.36	17.92±3.14	97.58±16.87	85.81±4.03	55.85±5.25	1.18±0.079
NS-m prior	100.31±21.60	12.27±3.04	62.76±6.81	88.34±4.61	59.14±6.79	1.23±0.038
after	122.38±40.57	35.80±7.38	127.21±12.02	72.11±6.47f	41.73±5.59e	1.20±0.028
NS-MI prior	109.57±11.57	11.87±1.04	103.78±14.13	89.19±1.47	59.94±2.21	1.19±0.032
after	353.45±79.49f	106.80±34.05f	317.49±21.58f	21.78±6.88f	42.06±11.53e	0.90±0.106f
RGE-b prior	121.52±18.87	10.16±0.59	112.13±11.78	91.39±2.08	63.65±3.86	1.21±0.039
after	142.19±17.56	22.23±2.07	80.6±4.46	84.08±4.29	53.88±5.31	1.20±0.025
RGE-m prior	131.47±15.97	23.27±1.44	100.52±8.95	82.29±1.45	51.44±1.63	1.24±0.084
after	108.9±37.43	32.59±4.62	174.89±22.25	69.55±5.76e	39.33±4.73	1.22±0.027
RGE-MIprior	117.11±29.94	21.65±7.55	100.00±19.54	83.29±9.09	53.55±9.83	1.23±0.147
after	338.28±47.84f	189.02±6.87f	260.61±32.38f	22.42±3.91f	43.08±6.28	0.89±0.086f

**Table 4:** UCE measurement before and 2 weeks after MI.

Group	LV,d (µl)	LV,s (µl)	LV,mass (mg)	LVEF (%)	LVFS (%)	E/A
NS-b prior	95.92±15.34	14.56±2.11	69.11±5.75	85.05±4.13	54.49±5.23	1.15±0.099
after	151.31±27.67	38.19±5.99	88.72±9.09	75.32±5.01	44.82±4.62	1.19±0.044
NS-m prior	106.00±8.63	15.48±1.29	71.18±6.89	85.32±2.80	54.76±3.60	1.19±0.067
after	127.51±22.59	32.56±8.79	100.00±24.94	75.67±9.87	45.51±9.14	1.13±0.041
NS-MI prior	83.21±31.23	9.06±4.14	60.87±4.86	90.26±5.37	61.91±7.77	1.27±0.048
after	342.60±28.62f	181.10±13.61f	301.18±21.07f	24.69±4.79f	46.94±7.82	0.83±0.076f
RGE-b prior	101.21±28.24	14.64±4.29	63.27±3.08	86.64±5.78	56.85±6.88	1.18±0.073
after	125.61±27.61	25.99±5.02	87.45±10.49	78.45±9.01	48.58±11.21	1.18±0.050
RGE-m prior	117.82±22.83	16.91±3.55	82.49±8.46	86.21±4.11	56.23±5.08	1.22±0.106
after	241.89±97.95f,g	88.00±21.25f,g	223.57±32.48f,h	65.66±7.43f	37.23±5.49e	1.17±0.086
RGE-MIprior	99.32±14.82	8.97±3.23	90.89±24.56	91.53±5.10	64.52±8.64	1.19±0.060
after	185.45±38.65h	98.34±16.13f,h	165.82±21.75h	47.18±9.97f,h	24.34±6.13f,g	0.91±0.026f

RETRACTED

**Table 5:** UCE measurement before and 4 weeks after MI.

Group	LV,d (µl)		LV,s (µl)	LV,mass (mg)	LVEF (%)	LVFS (%)	E/A
NS-b prior	104.31±38.15	16.59±4.70		87.28±11.29	85.57±5.65	55.52±6.91	1.21±0.048
after	161.26±30.61	41.51±6.66e		153.31±11.38	74.89±5.52e	44.57±5.24	1.15±0.046
NS-m prior	96.78±31.16	13.34±3.80		62.63±2.86	87.28±4.92	57.55±6.56	1.21±0.025
after	305.81±21.93e	116.11±5.58f		384.26±39.28f	62.03±3.06f	34.62±2.28f	1.19±0.050
NS-MI prior	89.44±15.05	9.06±1.95		64.68±8.50	89.98±3.58	61.19±5.97	1.20±0.053
after	347.4±23.18f	207.89±7.45f		264.27±23.91f	24.02±3.76f	35.52±14.58f	0.94±0.084f
RGE-b prior	99.67±44.15	10.21±2.10		76.88±10.05	89.11±3.46	59.88±6.10	1.19±0.027
after	125.21±18.79	30.26±4.55		84.37±8.84	76.30±6.34e	45.66±6.29e	1.18±0.042
RGE-m prior	93.36±7.21	9.32±0.95		69.33±4.20	90.04±1.78	61.96±1.88	1.19±0.038
after	184.4±41.21e,h	58.21±5.78f,h		143.40±14.32h	67.73±3.28e	38.41±2.83f	1.18±0.039
RGE-MI prior	100.60±41.53	7.51±1.30		80.78±11.92	92.23±1.65	64.67±3.40	1.20±0.079
after	169.03±22.4h	81.52±7.53f,h		135.40±10.19h	51.61±8.14f,h	26.98±5.04f	0.73±0.053f,h

LV-d, left-ventricular end-diastolic volume; LV-s, left-ventricular end-systolic volume; LV-mass, relative mass of left ventricle; LVEF, the left-ventricular ejection fraction; LVFS, the Left-ventricular fractional shortening; E/A, the radio of peak E velocity and peak A velocity at mitral valve protocol; NS-b, NS blank; NS-m, NS mock; RGE-b, RGE blank; RGE-m, RGE mock; prior, before MI; after, after MI and before being killed. Data are mean ± SD.

e P<0.05,

f P<0.01 vs. the same animal before MI;

g P<0.05,

h P<0.01 vs. blank group.

The significantly up-regulated serum levels of Tn-T and BNP in NS-MI and GRE-MI groups also showed the successful establishment of mouse MI model (P<0.01). After MI, the high level of Tn-T decreased in RGE group (from week 1, P<0.01 to 0.05) earlier than that in NS group (from week 4, P<0.01). As for BNP, the level increased from day 3 to week 4 with NS (P<0.01 to 0.05), while had no changes with RGE treatment after MI (Fig. 1-D). These revealed that RGE systemic delivery decreased myocardial damage and protected them from further inflammatory reaction after MI.

RETRACTED

Poley’s stain showed the ischemic myocardial zone (stained red) in normal myocardium (stained blue, Fig. 2-A). In chronic stage after MI, the relative ischemic area was lower with RGE than NS (P<0.05, Fig. 2-C). TUNEL stain and quantitative analysis showed that the apoptotic myocardium was less with RGE than NS in chronic stage after MI (P<0.01 to 0.05, Fig. 2-B, 2-C). These showed RGE’s function on improving ischemic myocardium and decreasing myocardial apoptosis.

**Figure 2:** Poley’s stain and TUNEL stain of ischemic myocardium. (A) Poley’s stain of NS-b, RGE-b, NS-MI, RGE-MI groups at week 4. The ischemic areas were stained red indicated by red arrow and non-ischemic area were stained blue. (B) TUNEL stain of NS-b, RGE-b, NS-MI, RGE-MI groups at week 4. The apoptotic myocardial cells were green under fluorescent and brown under Immunohistochemistry stain indicated by red arrow. (C) Quantitative analysis of mean relative ischemic area (percentage of the total transverse sections area) and myocardium apoptotic index (ratio to total myocardial cells). Data are mean ± SD. *P<0.05, **P<0.01 vs. NS group at the same time, ^#^P<0.05, ^##^P<0.01 vs. the same group at day 3, ^$^P<0.05, vs. the same group at week 1.

### RGE’s Function on Activating EPCs

EPCs were identified as Dil-acLDL and FITC-UEA-1 double-stained cells with the nuclei stained by DAPI (Fig. 3-A). FACS was used to analyze the quantity of EPCs marked by CD34, VEGFR2 and CD133 in blood and bone marrow (Fig. 3-B).After MI, the quantity of EPCs in peripheral blood increased (P<0.01) and it decreased in bone marrow (P<0.05) with both RGE and NS. These suggested that the EPCs in bone marrow were mobilized to peripheral blood as the injury of myocardium. In chronic stage after MI, the increase of EPCs in peripheral blood was more significant with RGE compared to NS (P<0.01), and the decrease of EPCs in bone was not so much with RGE as it with NS (Fig. 3-C). These suggested that in chronic stage after MI, RGE was able to increase EPCs mobilizing to ischemic myocardium and maintain the quantity of EPCs stored in bone marrow. With the increased EPC population in both bone marrow and peripheral blood, the total number of EPCs in vivo was much more with RGE than NS.

**Figure 3:** Effect of RGE on endothelial progenitor cells (EPCs) number. (A) EPCs were identified by Dil-acLDL (red), lectin-FITC (green) and DAPI (blue) staining. (B) FACS analysis of peripheral blood and bone marrow levels of EPCs with 3 surface markers: CD34-PE, VEGFR2-FITC, CD133-PerCP-Cy5.5 at week 4. (C) Quantification of percentage of triple-marked cells from the initial monocytes in gate. Data are mean ± SD. *P<0.05, **P<0.01 vs. NS group at the same time, ^#^P<0.05, ^##^P<0.01 vs. the same group at day 3.

RETRACTED

By MTT assay, we tested the proliferation of EPCs in each group. The MI surgery made the proliferated activity of EPCs up-regulated with both GRE and NS (P<0.01). However, it maintained at a high level with RGE compared to it decreased in week 2 and 4 with NS (P<0.05, Fig. 4-A). These showed that RGE was able to up-regulated the proliferation of EPCs after MI, especially in chronic stage. At week 4 after MI, the migration of EPCs was more active with RGE than NS (P<0.05, Fig. 4-B, 4-D). From week 2 after MI, EPCs participated in capillary-like tube formation were increased with RGE compared to NS (P<0.05), and a similar increase occurred in normal rats with RGE relative to NS (P<0.05, Fig. 4-C, 4-D). These suggested REG’s function on motivating EPCs tube-formation capacity after MI as well as in normal physiological status.

**Figure 4:** Effect of RGE on EPC function. (A) MTT assay of proliferation of EPCs. (B) Transwell-chamber migration assay of EPCs at week 4. The activated EPC (marked by red arrow) migrated from upper chamber to the lower chamber. (C) Assessment of angiogenesis with EPCs placed on Martrigel and forming tubular-like structures at week 2. EPCs integrated in tubular-like structures are marked by red @; the formed tube was marked by red arrow. (D) Quantification of migration and angiogenesis of EPCs. For migration, data are percentage of EPCs migrating to the lower chamber as compared with those in the upper chamber. For angiogenesis, data are the ratio of EPCs integrated in tubular-like structures and the tubes involved. Each test was repeated 4 times, and data are mean ± SD. *P<0.05 vs. NS group at the same time, ^#^P<0.05 vs. the same group at day 3.

### RGE’s Function on Therapeutic Angiogenesis

Immunohistochemistry showed the fluctuant expression of VEGFR2 and CD133, which were signals of new-born capillary. After MI, the expression of VEGFR2 increased from week 1 until week 4 with RGE (P<0.05 to 0.01), and was much more significant than that with NS (P<0.05 to 0.01). In chronic stage after MI, the expression of CD133 also increased more with RGE than NS (P<0.01, Fig. 5-A, 5-B). The expression fluctuation at the level of mRNA was almost the same (Fig. 5-C). These revealed that RGE was able to promote the newborn of capillary at the chronic stage of MI.

**Figure 5:** Effect of RGE on angiogenesis at the MI area. (A) Immunohistochemistry of VEGFR2 and CD133 in NS-b, NS-MI, RGE-b and RGE-MI groups at week 4. The vessels are indicated by red @, and positive colorations are indicated by red arrows. (B) Quantification of VEGFR2 and CD133 immunoreactivity (percentage of positive area) in each group. (C) Quantitative PCR analysis of VEGFR2 and CD133 in myocardial tissue. For real-time PCR, the NS-b group was considered the baseline, actin was the internal reference. Data are mean ± SD. *P<0.05, **P<0.01 vs. NS group at the same time, ^#^P<0.05, ^##^P<0.01 vs. the same group at day 3, ^$^P<0.05, ^$$^P<0.01 vs. the same group at week 1.

RETRACTED

### RGE’s Function on SDF-1α/CXCR4 Cascade

To investigate the mechanism involved in effect of RGE on EPCs, we detected the change in SDF-1α/CXCR4 cascade expression with MI in vivo, and with cellular experiments in vitro.

Immunohistochemistry revealed the increased protein expression of CXCR4 in MI groups compared to control groups (P<0.01) and the increase was more significant with RGE than NS in chronic stage after MI (P<0.01, Fig. 6-A, 6-B). Western blots analysis revealed the same findings for CXCR4 protein expression in ischemic myocardial tissue. As for SDF-1α, the expression increased with RGE but not with NS at week 1 compared to day 3 (P<0.01). And there was no statistical difference between the two treatments in chronic stage after MI (Fig. 6-C, 6-D). RT-PCR showed the changes in mRNA level of SDF-1α/CXCR4 cascade. The fluctuation of mRNA expression was just like what it showed in protein expression by Western blot (Fig. 6-E). These suggested that RGE might activate SDF-1α/CXCR4 cascade mainly by up-regulating transcription and translation of CXCR4.

**Figure 6:** The expression of the stromal-derived factor-1α (SDF-1α) and its receptor 4 (CXCR4) in tissue. (A) Immunohistochemistry of CXCR4 in NS-b, NS-MI, RGE-b and RGE-MI groups at week 4. The vessels are indicated by red @, and positive colorations are indicated by red arrows. (B) Western blot analysis of protein expression of CXCR4 and SDF-1α. β-actin was an internal reference protein for Western blot. (C) Quantitative of CXCR4 immunoreactivity (percentage of positive area) in each group. (D) Quantitative Western blot analysis of CXCR4 and SDF-1α in myocardial tissue. (E) Quantitative PCR analysis of CXCR4 and SDF-1α in myocardial tissue. Data are mean ± SD. *P<0.05, **P<0.01 vs. NS group at the same time, ^#^P<0.05, ^##^P<0.01 vs. the same group at day 3, ^$^P<0.05, ^$$^P<0.01 vs. the same group at week 1.

To further certify the effect of RGE on SDF-1α/CXCR4 cascade, EPCs were stimulated with RGE-PBS solutions in vitro. The proliferation of EPCs decreased with 500 and 1000 µg/ml RGE solution (Fig. 7-A), so we chose other 4 kinds of solutions (10, 25, 50, 100 µg/ml) in subsequent experiments. Through Western blot and RT-PCR, we chose the optimal RGE-PBS solution concentration and duration for SDF-1α/CXCR4 cascade (Fig. 7-B to 7-E). For CXCR4, the optimal concentration is 25 µg/ml (P<0.01) and the optimal duration is 48 h (P<0.05 to 0.01). For SDF-1α, the optimal concentration is 50 µg/ml (P<0.01) and the optimal duration is 24 h (P<0.01). The optimal concentration and duration were used to stimulate EPCs and the tube-formation capacity of EPCs was tested. The inhibitor group, blocking the SDF-1α/CXCR4 cascade with AMD3100, showed poor functional EPCs that barely participated in capillary-like tube formation, CXCR4 showed poor expression and its ligand SDF-1α showed over-expression (P<0.01). The CXCR4 optimal concentration and duration (RGE = 25 µg/ml, 48 h) most significantly increased EPCs participating in capillary-like tube formation as compared with the other groups (P<0.05 to 0.01). The optimal concentration and duration for SDF-1α (RGE = 50 µg/ml, 24 h) had a similar but not as obvious an effect as for CXCR4 (P<0.05 to 0.01). These revealed that RGE was able to increase EPCs participating in capillary-like tube formation by up-regulating SDF-1α/CXCR4 cascade expression in vitro. And this effect of RGE could be reversed by CXCR4 specific inhibitor AMD3100.

**Figure 7:** Effect of RGE on SDF-1α/CXCR4 cascade in vitro. (A) MTT assay for proliferation of EPCs after stimulation with RGE-phosphate buffered saline (PBS) solutions. The final concentration of RGE-PBS solution was 10 µg/ml (RGE = 10), 25 µg/ml (RGE = 25), 50 µg/ml (RGE = 50), 100 µg/ml (RGE = 100), 500 µg/ml (RGE = 500) and 1000 µg/ml (RGE = 1000). (B) Western blot analysis of protein expression of SDF-1α/CXCR4 cascade with EPCs treated by different concentrations of RGE-PBS solutions. (C) Western blot analysis of protein expression of SDF-1α/CXCR4 cascade with EPCs stimulated for different times. (D) Expression of SDF-1α/CXCR4 cascade in EPCs with RGE treatment. The final concentration of RGE-PBS solution was 100, 50, 25 and 10 µg/ml. The duration of stimulation was 72 h. Control, culture with only EBM-2. Inhibitor, pre-stimulated with specific CXCR4 antagonist AMD3100 (5 µg/ml) for 1 h, then with RGE (100 µg/ml, 72 h). (E) Expression of SDF-1α/CXCR4 cascade with EPCs stimulated for different times. The final concentration of RGE used to stimulate EPCs was 25 µg/ml for CXCR4 and 50 µg/ml for SDF-1α. Control, culture with EBM-2 without RGE for 72 h. RGE groups, stimulation for 6, 12, 24, 48 and 72 h. (F) EPCs’ tube-formation capacity in vitro. C, control group culture with only EBM-2. AMD, pre-stimulation with AMD3100 (5 µg/ml) for 1 h and then RGE at 25 µg/ml for 48 h. RGE25-48 h, RGE at 25 µg/ml for 48 h. RGE50-24 h, RGE at 50 µg/ml for 24 h. Data are ratio of EPCs integrated in tubular-like structure (marked by red @) and the tubes involved (marked by red arrow). Each test was repeated 3 times and every group had 3 repetitive wells on one 6-well plate. Data are mean ± SD. *’P<0.05, *P<0.01 vs. all the other groups.

RETRACTED

## Discussion

The traditional Chinese herb Rehmannia glutinosa can promote bone-marrow proliferation and protect the ischemic myocardium without mechanism studied [15], [16]. And the EPCs are attractive targets for repair of the ischemic myocardium [1]–[3]. Therefore, we investigated the effect of RGE on EPCs in a rat model of MI. In preliminary experiments, 3 different oral doses of RGE given to normal rats could increase the number of EPCs in peripheral blood and bone marrow at 8th to 16th weeks. Among these, the high dose had the most significant effect at 8th to 12th weeks (P<0.01; TableS1). The preliminary experiment showed that the RGE made effect on EPCs needed a relatively long time (about 12 weeks). And the mortality of rats after MI will increase with the time goes by. So we orally fed high-dose RGE (1.5 g·kg-1·day-1) to rats 8 weeks before MI induction and 4 weeks after MI. RGE significantly improved ischemic myocardium and protect left ventricular function after MI. As well, RGE activated EPCs by promoting their proliferation, mobilization, migration and participating in therapeutic angiogenesis at the ischemic region. It also up-regulated the expression of angiogenesis-associated ligand/receptor CD133, VEGFR2, SDF-1α and CXCR4. As these effects of RGE almost occurred at the chronic stage after MI (systemic delivered for 10 to 12 weeks), we suggested that patients with MI might benefit from RGE in chronic stage rather than acute stage. RGE could be an EPC activator mediated by SDF-1α/CXCR4 cascade activation, thus preserving the ischemic myocardium in rats.

The changes showed in ECG, UCG and significant increased Tn-T, BNP level revealed the successful establishment of the MI model, with no difference between NS and RGE in 3 days after MI. Thus, RGE might not produce effects in a relatively short time. RGE began to have effects in the chronic stage of MI (from weeks 2 to 4). In the chronic stage after MI, the LV-mass was lower with RGE than NS because of the decreased LV-d and LV-s, the LVEF and LVFS were higher with RGE than NS, although still less than those in the blank and mock groups. RGE ameliorated the MI-induced Tn-T increasing before the NS effected and prevented the BNP level from increasing as with NS. The relative ischemic area and myocardial apoptotic index in the infarcted myocardium was decreased with RGE than with NS. Therefore, at the chronic stage of MI, RGE could preserve the ischemic myocardium by enhancing the function of the left ventricle, decrease the risks of acute coronary syndromes associated with increased BNP [30] and apoptosis in the myocardium.

RETRACTED

To determine whether the RGE’s effects on ischemic myocardium are associated with its effects on EPCs showed in preliminary experiments, we examined the number and function of EPCs obtained from peripheral blood and bone marrow of rats. Stem cells, including EPCs, can be mobilized from the bone marrow and other niches, homing to the area of injured tissue and trans-differentiating into functional cardiomyocytes [4]–[5], [31]–[32]. Here we defined EPCs as cells that can absorb ac-LDL and UEA-1 [23] and counted the number of cells positive for CD34, CD133 and VEGFR2, widely accepted markers of EPCs [33]–[35]. In peripheral blood, the number of EPCs increased in acute stage after MI and it went on increasing with RGE but not NS in the chronic stage. In bone marrow, the EPC number decreased with NS because of EPCs mobilizing from bone marrow to blood, while it maintained high with RGE. The increase in RGE-b and RGE-m groups compared with respective NS groups coincided with our preliminary study. In the chronic stage of MI, RGE statistically activated EPC function as compared with NS: in increased EPCs proliferation, migration and tube-formation capacity. These effects occurred later after MI, especially for migration made effect until week 4, might attribute to multitudinous EPCs migration occurred at the terminal stage of acute cardiovascular event and the slow-release of RGE. In general, RGE could increase the number of EPCs in normal and MI rats by increasing the storage in bone marrow and increasing the mobilization to peripheral blood, then migration to injured tissue. Besides increasing cellular number, RGE also activated the function of EPCs, which made them available for the injured myocardium.

Angiogenesis is the most important way to improve the supply of blood to the infarcted myocardium and an important potential role for EPCs, especially for development of new capillaries in adults [36]–[38]. The detection of new capillaries may be an effective way to explain the relationship between the effect of RGE on the infarcted myocardium and on EPCs. CD133 and VEGFR2, markers of EPCs which participated in new-born capillary, are also effective markers of early stage angiogenesis [33]–[36]. We tested the levels of thm in infarcted tissue to reflect the level of angiogenesis. The expressions of CD133 and VEGFR2 were greater with RGE than NS at the chronic stage of MI. From these we suggested that RGE activated the EPCs with CD133 and VEGFR2 migrating to ischemic region, then increased them participated in capillary-like tube formation, and further developed to new-born capillary which highly expressed CD133, VEGFR2. Therefore, RGE is able to increase new-born capillary formation. Combined with RGE’s effect on increasing the number and function of EPCs, RGE protect the myocardium after MI through angiogenesis mediated by EPCs.

RETRACTED

The expression of the SDF-1α/CXCR4 cascade was increased with RGE after MI. SDF-1α–CXCR4 interaction plays a crucial role in recruiting EPCs to the heart after MI and could increase homing, thus inducing border-zone angiogenesis and preserving ventricular function [12]–[13]. We observed this effect of RGE on the SDF-1/CXCR4 cascade after MI, the expression of CXCR4 was up-regulated while there was no statistic different in SDF-1α expression. When SDF-1α reactive with CXCR4, Arg8 and Arg12 of SDF-1α bind with Glu15 and Asp20 of CXCR4 firstly, and make the disruption of the salt bridge between Arg188 and Glu277 in CXCR4, then Lys1 of SDF-1α bind with Asp262 which was exposed from the disrupted salt bridge in CXCR4, in this way activate SDF-1α/CXCR4 cascade and signal transduction down-stream [39], [40]. Thus, we suggested that RGE activated SDF-1α/CXCR4 cascade mainly through increasing the expression of CXCR4 and activating SDF-1α/CXCR4 interaction mediated by CXCR4, then the EPCs were mobilized and homing to the injured region [9], [13]. In this way, the SDF-1α/CXCR4 cascade was involved in mediating RGE’s effects. To confirm our finding and search for the therapeutic theory of RGE, we used RGE-PBS solution to stimulate EPCs in vitro. The expressions of both SDF-1α and CXCR4 were higher with RGE than the control group. RGE was able to up-regulate tube-formation capacity of EPCs at its optimal actuation concentration and duration. When stimulated with RGE at its optimal actuation concentration and duration for CXCR4 and SDF-1α, the tube-formation capacity of EPCs was up-regulated. When SDF-1α/CXCR4 was blockade by specific CXCR4 inhibitor AMD3100, RGE had no effect on EPCs, CXCR4 showed poor expression and its ligand SDF-1α showed over-expression. Therefore, RGE promoted EPCs function by up-regulating the expression of the SDF-1α/CXCR4 cascade, and with the SDF-1α/CXCR4 cascade blocked, the effects of RGE were eliminated. RGE may mobilize EPCs in bone marrow and for migration to the injured myocardium, thus enhancing local angiogenesis after MI, with the SDF-1α/CXCR4 cascade involved in mediating RGE’s effects on EPCs after MI.

Although RGE was alcohol extracted from the herb Rehmannia glutinosa, the specific structures and molecular formulas of RGE remain to be clarified. As well, we certified that the activation of SDF-1α/CXCR4 cascade was involved in mediating RGE-associated EPC activation after MI, but the detailed genetic loci underlying require further investigation.

RETRACTED

In summary, we demonstrated that in rats with MI, extracts of the herb Rehmannia glutinosa promoted the mobilization of EPCs in bone marrow, enhanced their migration to the local ischemic region and participation in angiogenesis, thus preserving the ischemic myocardium. The mechanism may involve mediation by the SDF-1α/CXCR4 cascade.

## Supporting Information

Table S1 **Effect of RGE on endothelial progenitor cell (EPC) number.** Control, rats oral-treated with normal saline (NS); RGE-L, rats oral-treated with RGE at 0.38 g·kg^−1^·day^−1^; RGE-M, rats oral-treated with RGE at 0.75 g·kg^−1^·day^−1^; RGE-H, rats oral-treated with RGE at 1.5 g·kg^−1^·day^−1^. Data are mean ± SD. ∧P<0.05, *P<0.01 vs. control group.
(DOCX)
